# Improved Cellular Specificity of Plasmonic Nanobubbles versus Nanoparticles in Heterogeneous Cell Systems

**DOI:** 10.1371/journal.pone.0034537

**Published:** 2012-04-03

**Authors:** Ekaterina Y. Lukianova-Hleb, Xiaoyang Ren, Pamela E. Constantinou, Brian P. Danysh, Derek L. Shenefelt, Daniel D. Carson, Mary C. Farach-Carson, Vladimir A. Kulchitsky, Xiangwei Wu, Daniel S. Wagner, Dmitri O. Lapotko

**Affiliations:** 1 Department of Biochemistry and Cell Biology, Rice University, Houston, Texas, United States of America; 2 Department of Clinical Cancer Prevention, The University of Texas MD Anderson Cancer Center, Houston, Texas, United States of America; 3 Institute of Physiology, National Academy of Science of Belarus, Minsk, Belarus; 4 Department of Physics and Astronomy, Rice University, Houston, Texas, United States of America; University of Notre Dame, United States of America

## Abstract

The limited specificity of nanoparticle (NP) uptake by target cells associated with a disease is one of the principal challenges of nanomedicine. Using the threshold mechanism of plasmonic nanobubble (PNB) generation and enhanced accumulation and clustering of gold nanoparticles in target cells, we increased the specificity of PNB generation and detection in target versus non-target cells by more than one order of magnitude compared to the specificity of NP uptake by the same cells. This improved cellular specificity of PNBs was demonstrated in six different cell models representing diverse molecular targets such as epidermal growth factor receptor, CD3 receptor, prostate specific membrane antigen and mucin molecule MUC1. Thus PNBs may be a universal method and nano-agent that overcome the problem of non-specific uptake of NPs by non-target cells and improve the specificity of NP-based diagnostics, therapeutics and theranostics at the cell level.

## Introduction

Nanomedicine promises unique abilities to support diagnostic, therapeutic and theranostic functions at nanoscale, providing molecule- and cell-level resolution, specificity and selectivity. These functions are usually mediated through nanoparticles (NPs) that have to be delivered to specific molecular and cellular targets associated with a certain pathology or diagnosis. However, this strategic advantage of nanomedicine is compromised by the principal limitation in NP targeting. This is that no current method can deliver NPs only to target cells and molecules because some amount of NPs always accumulates non-specifically in non-target cells, thus reducing the specificity and selectivity of nanomedicine. The limited specificity of NP targeting, in turn, requires higher loads of NPs in order to achieve the desired diagnostic or therapeutic effect [1]–[8]. The high loads of NPs required for therapy delivery further induces non-specific accumulation and cause toxicity issues because most NPs are inorganic and of non-biological origin. Increased NP loads and low targeting specificity result in macro- rather than nano-resolution for NP medicines. Among NPs, those based on gold have been exploited most often. Gold NPs have low toxicity [9], [10] and have been used in a relatively wide spectrum of biomedical applications: optical [6], [11]–[13] and photoacoustic [14], [15] diagnostics, drug delivery [12], [16]–[19], the direct destruction of target cells through photothermal effects [1]–[7], [20]–[29], or in combination with chemotherapy [30]. In addition, gold NPs were applied in combination with other NPs such as drug carriers and diagnostic labels [31]–[37].

The specificity of NP targeting to specific (target) cells was improved by chemically attaching target-specific vectors to the gold NPs thus coupling NPs to specific target receptors at cellular membrane [12], [38]–[47]. This active targeting is more effective compared to passive targeting with “bare” non-functionalized NPs. However, many cellular receptors are widely expressed, albeit at very different levels, on target and non-target cells (bio-heterogeneity). As a result, a considerable number of actively targeted NPs will still get to non-target cells through various non-specific mechanisms [1]–[7]. Therefore, the targeting of NPs to cells so far cannot provide sufficient specificity, which slows the translation of nanomedicine to clinic.

The high biomedical specificity of NP-based effects could be achieved by activating them with a *threshold mechanism* that would efficiently discriminate between NPs in target and non-target cells. These effects are optical scattering, fluorescent and photoacoustic diagnostics, drug delivery and release, and photothermal therapeutics. Most of the current methods activate these NP effects in cells in a linear way without a threshold effect and thus such methods often cannot discriminate between target and non-target cells.

Recently we demonstrated a novel cell-level transient nano-phenomenon, the plasmonic nanobubble (PNB). This transient nano-event is triggered by the short pulsed optical heating of gold NPs and has a threshold of generation that is sensitive to multiple variables including clustering of NPs [48]–[51]. A PNB is a vapor nanobubble transiently induced around a superheated gold NP upon its activation with a short laser pulse whose energy is converted by the gold NP into heat through the mechanism of plasmon resonance [3]–[5], [12], [13], [49], [52], [53]. PNB generation threshold energy was found to depend upon NP structure, size and aggregation state and was found to be lowest for NP clusters, nanostructures with tightly aggregated NPs [48], [54], [55]. This unique physical property of PNBs allows their selective generation under low laser pulse fluence only around large clusters of NPs, while the same level of laser fluence was below PNB generation threshold for single NPs or their small clusters. As biomedical agents, PNBs demonstrated their potential for optical diagnostics [40], [56]–[58], delivery and on demand release of therapeutic and genetic cargo [59]–[62], elimination of target cells [38], [49], [63], [64], microsurgery [65], [66] and theranostics [40], [55], [63].

We hypothesized that combining the threshold nature of gold NP-generated PNBs with their biomedical properties could significantly improve the precision and specificity of gold NP-based biomedical effects (Figure 1). Despite extensive previous studies of PNBs and especially of gold NPs in cells, validation of this hypothesis requires direct comparison of the specificity of NPs and PNBs in target vs non-target cells, a study that has not occurred. To validate this hypothesis we compared the abilities of PNBs and gold NPs to discriminate between target and non-target cells under identical treatment conditions in six different *in vitro* models and molecular targets. We demonstrate an efficient and universal solution for overcoming the influence of non-specific accumulation of NPs in non-target cells and to achieve high cellular specificity of biomedical effects of NPs.

**Figure 1:** PNBs and NPs in target (left panels) vs non-target (right panels) cells. A: gold NP conjugates are collected at cellular membranes and are clustered during endocytosis resulting in the largest NP clusters in target cells. B: Excitation laser pulse (green) of low fluence induces PNBs only around the largest NP clusters (i.e. only in target cells) because the PNB generation threshold fluence for single NPs and small clusters (non-target cells) is higher than the fluence of the laser pulse. C: Optical scattering of the probe laser radiation (red) by PNBs provides its real-time imaging and monitoring in the individual cell (ID: image detector, RD: response detector).

## Methods

### 1. Nanoparticles and their clusters

We have used three different types of gold nanoparticles (NP): commercially available 60 nm spheres (NSP) and fabricated 50 nm hollow gold nanoshells (NS) and 110 nm gold NS with silica core inside. Gold NSP were provided and conjugated with cell-specific antibodies by Bio Assay Work LLC (Ijamsville, MD). 50 nm hollow gold NSs were synthesized by galvanic replacement of gold on a silver core according to Zasadzinski et. al. [67] The advantages of this type of NP include low toxicity, reliable conjugation properties, relatively high photothermal efficiency and maximal plasmonic nanobubble (PNB) generation efficacy in the biologically safe near-infrared spectral region with reducing the PNB generation threshold laser fluence. The 110 nm gold NS with silica core inside were designed and fabricated as described in previously [4]. NSs structure and size were verified with TEM (JEOL 2010, Jeol Ltd., Tokyo, Japan). Optical density spectra of NPs were obtained in water with a spectrophotometer (the USB 650 Red Tide spectrometer, Ocean Optics, Inc, Dunedin, FL).

For the study of PNB generation around NP clusters in water, NS clusters were prepared by adding sodium chloride to a suspension of single NSs. Clusters were re-suspended in water to provide low surface density that provided exposure of only one NP cluster by a single laser pulse. Next, we added 5 µl polysterene microspheres of 7.6 µm diameter (Spherotech Inc., Lake Forest, IL) were added into 50 µl of the NS clusters suspension. These microspheres have been used as spacers between the two glasses (a standard microscope slide and coverslip of 18 mm diameter) to provide a specific height (7.6 µm) of the sample volume. Clusters were re-suspended in water so that their low surface density would exclude the exposure of closely located nanoparticles under laser irradiation. To minimize the effect of cluster size heterogeneity, we used only the clusters with close levels of pixel image amplitudes of their optical scattering images. Each cluster was positioned in the center of the excitation laser beam and was exposed to a single laser pulse.

### 2. Molecular targets and cell models

We studied the six cell models representing four molecular targets (Table 1). Each pair of cells represented target cells with high level of expression of specific molecular target and non-target cells with low level of the expression of such molecular target. Details on culturing cells and monitoring of the expression level of molecular targets can be found in Text S1 and Figure S1 and Figure S2. NP clusters were selectively formed in target cell though the two-stage mechanism (Figure 1a):

at the first stage we used target-specific antibodies to provide higher accumulation of gold NPs at the membranes of target cells compared to the NP accumulation at membranes of non-target cells. This stage did not provide desired specificity of the targeting but at the same time delivered much more NPs to target cells compared to non-target cells;
at the second stage we engaged receptor-mediated endocytosis so that target cells self-assembled the large clusters of gold NPs in their endosomal systems [38]–[46].

**Table 1:** Cell models and conditions of their treatment with NP and laser pulses.

				Incubation conditions		Laser pulseparameters		
Mole-cular target	NP	Vector	Cells:target/non-target	NP con-centratio, NP/ml	Incu-bation time	Dura-tion, ps	Wave-length, nm	Fluence, mJ/cm^2^
EGFR	50 nmNS	Panitu-mumab	HN31/NOM9	2.4*10^10^	24 h	70	820	30
EGFR	60 nmNSP	Panitu-mumab	HN31/NOM9	2.4*10^10^	24 h	70	532	60
EGFR	60 nmNSP	C225	HN31/NOM9	2.4*10^10^	24 h	70	532	60
-	60 nmNSP	none	HN31/NOM9	2.4*10^10^	24 h	70	532	60
EGFR	110 nmNS	C225	C42B/HS5	1.2*10^11^	30 min	500	787	38
MUC1	60 nmNSP	214D4	HES/HS5	2.4*10^10^	1 h	500	532	40
PSMA	60 nmNSP	Anti-PSMA	C42B/HS5	1.2*10^11^	30 min	500	532	60
CD3	60 nmNSP	OKT3	CD3+ T-cells/CD3− BMC	1.2*10^11^	30 min	70	532	37
CD3	60 nmNSP	OKT3	J32/JRT3-T3.5	1.2*10^11^	45 min	500	532	63
EGFR	60 nmNSP	C225	A549/Fibro-blasts	6*10^10^	30 min	500	532	30

The targeting parameters such as the concentration of NPs and the incubation time were optimized to achieve maximal difference in NP uptake between the target and non-target cells (Table 1). Applied targeting method does not eliminate the non-specific uptake of NPs, however, it provides the formation of the largest NP clusters only in target cells for target-specific generation of PNBs. Table 1 resumes experimental conditions applied for each molecular target and cell model. Sphere- and shell-type NP conjugates did not induce any considerable cytotoxicity in either target or non-target cells within 48–72 h (see Supplementary Information for details). Both cell cultures were identically treated with NPs conjugated to target-specific antibodies.

### 3. Generation of plasmonic nanobubbles

PNBs were generated due to transient heating of gold NPs with single laser pulses to the temperatures well above the evaporation threshold for the liquid environment of NPs (Figure 1b). We employed single short laser pulses of 70 and 400 ps, 532 nm (for excitation of solid gold spheres) and 787 nm (for excitation of gold nanoshells) (PL-2250, Ekspla and and STH-01, Standa Ltd, Vilnius, Lithuania). A short laser pulse maximized the efficacy of NP heating by preventing three negative processes: thermal losses through thermal diffusion [68], NP photodamage [69] and attenuation of incident optical pulse by developing vapor bubble [70]. Such vapor nanobubble uses thermal energy generated by gold NPs through the mechanism of plasmon resonance [3]–[5], [12], [13], [49], [52], [53] and this thermal energy (1) determines maximal diameter and lifetime of PNB and (2) is determined by fluence of laser pulse [54], [55]. Fast adiabatic expansion of the PNB provides efficient thermal insulation of its environment from the internal heat [54], [71]. The described mechanism also explains the origin of the term “plasmonic nanobubbles”: such vapor bubbles get their energy through plasmon resonance of gold NPs and act at nanoscale as mechanical, optical and acoustic nano-agents. Optical generation and detection of the PNBs was performed with a photothermal laser microscope that we developed previously [40], [48]. The laser pulse fluence (10–90 mJ/cm^2^) was experimentally determined for each pair of the target and non-target cells to exceed the PNB generation threshold in target cells and to be below PNB generation threshold for non-target cells (see also Text S1 and Figure S3).

### 4. Optical detection of NPs and PNBs

To image and quantify the uptake of gold NPs by cells we imaged and measured optical scattering by gold NPs in individual cells. Amplitude of optical scattering signal correlates to the size of scattering nanoobject [54], [56] even if the latter is below optical diffraction limit and cannot be seen in a microscope. As a rule we used laser confocal microscopy (LSM 710, Carl Zeiss Microimaging Inc., Germany) to obtain the stack of several images per each cell (in case of A549 cells the NP scattering was imaged and quantified with regular inverted microscope). In each population (sample) 30–50 cells were analyzed and the population-average image pixel amplitudes were calculated for each cell sample. Excellent optical scattering properties of a PNB [54] were used for its imaging in water and cells (Figure 1c) with two probe laser beams, pulsed probe beam (576 nm, 70 ps, 0.1 mJ/cm^2^) and continuous probe laser (633 nm). This provided two independent signals and two optical metrics of PNB (Figure S3): optical scattering time-resolved image pixel amplitude and duration of optical scattering time response (measured independently and simultaneously with optical scattering image). First, time-resolved optical scattering was used for imaging of PNBs and analyzing of their brightness. The maximum pixel amplitude of PNB was used as PNB metric (see Text S1 detailed definitions). The second PNB metric was independently obtained with another, continuous, probe laser (Figure S3). The PNB-induced scattering of a part of the probe beam decreased its axial amplitude, resulting in a dip-shaped output signal of the photodetector that monitored the probe beam. Thus we registered the time response of the probe laser radiation to the transient scattering effect of the PNB. This mode provided the monitoring of PNB growth and collapse, and delivered the PNB lifetime that characterizes its maximal diameter [23], [24], [48], [54], [55]. All three described above metrics were obtained for individual cells and were averaged for each population of target and non-target cells. This provided maximal precision of NP and PNB analysis.

## Results

### 1. The PNB creates a threshold response to the optical excitation of gold NPs

The physical mechanism of PNB specificity was studied by generating and analyzing single PNBs around individual gold NP clusters of variable size in water. NP clusters were prepared by aggregating gold NPs (hollow gold 50 nm nanoshells) in a high salt solution. We used single and clustered gold spheres (60 nm) and hollow shells (50–60 nm) (see Text S1 for details). Optical scattering imaging of NP clusters was used to characterize their size through the scattering image amplitude since optical scattering brightness correlates to the size of the scattering object [20], [72]–[74]. PNBs were detected around specific individual NP clusters with two simultaneous techniques, time-resolved optical scattering images and time response (see Text S1). Three PNB parameters, these being the probability of PNB generation, scattering image amplitudes and time response durations, were measured for individual PNBs as functions of the optical fluence of the excitation laser pulse and the brightness of the NP cluster. The excitation fluence that corresponded to the probability of PNB generation of 0.5 was defined as the PNB generation threshold. First we studied the dependence of the PNB threshold in a single pulse mode upon NP cluster size, measured through its scattering image amplitude (Figure 2a). We observed a significant reduction of the threshold fluence with the NP cluster size. Thus a low fluence was sufficient to generate PNBs around large NP clusters but was not sufficient to induce PNBs around single NPs or small NP clusters. This was demonstrated by exposing multiple NP clusters of various sizes to a single laser pulse of low fluence. We observed the selective generation of PNBs only around the largest NP clusters (Figure 2b) whose threshold was lower than the applied fluence. The PNB threshold for smaller clusters was above this fluence and, therefore, such small NP clusters did not return PNBs in response to optical excitation.

**Figure 2:** Parameters of PNBs generated around gold NP clusters in water for gold nanoshells. A: PNB generation threshold fluence of the excitation laser pulse as function of NP cluster size (measured through optical scattering amplitude of NP cluster image for individual clusters); B: PNB lifetime and scattering brightness as function of the NP cluster size (measured through optical scattering amplitude of NP cluster image) at specific fluence of the excitation pulse (778 nm, 22 mJ/cm^2^).

The dependence of the PNB threshold fluence upon cluster size can be explained through the mechanism of PNB generation around superheated NPs. Merged thermal fields of several tightly aggregated NPs form a common thermal field and vapor layer around the cluster. The initial vapor pressure in such a vapor layer is determined by the fluence of the laser pulse that is converted into heat by each NP in a cluster. Next, the external pressure of surface tension (that needs to be overcome to allow the expansion of the vapor) is inversely proportional to the radius of the vapor-liquid boundary [75]–[77] and, therefore, decreases with cluster size. We previously analyzed the mechanism of PNB generation around NP clusters versus single NPs [54]. In addition to the above thermal and hydrodynamic factors, NP clustering may enhance their optical absorbance [78], [79], thus additionally increasing the released thermal energy and the initial vapor pressure. All these factors cause the decrease of the PNB generation threshold fluence with cluster size. With the fluence of the excitation pulse below the threshold, the PNB does not emerge, and, therefore, creates no impact, unlike NPs (Figure 2b). Contrary to a gradual increase in optical scattering amplitude of NP clusters with their size, the PNB scattering signals responded to a threshold NP cluster size (Figure 2b). This resulted in the selective generation of PNBs only around the largest NP clusters, while no PNBs emerged around single NPs and small clusters under identical excitation conditions. This cluster-threshold mechanism of PNBs created a unique opportunity to improve the specificity of NP-based effects.

### 2. Cellular specificity of NPs and PNBs

Since the largest NP clusters can be selectively formed in target cells through the receptor-medicated endocytosis of NPs [38]–[46], we further studied the NP cluster-PNB mechanism in living cells in order to compare the cellular specificity of NPs and PNBs under identical conditions of NP targeting and optical excitation. Several different molecular targets were investigated *in vitro* in cell systems that included cells with a high level of molecular target expression (target cells) and a low level of the expression of the same molecular target (non-target cells).

We studied cell models representing lung (A549), head and neck (HN31), prostate (C4-2B), epithelial (HES, a WISH/HeLa derivative) and blood (Jurkat J32) cancers and also human T-cells that are used for gene therapies of cancer (see the detailed description of experimental models in Text S1). Both solid gold spheres (NSP) and gold nanoshells (NS) were conjugated to target-specific antibodies (Table 1, see also Text S1) and were administered under concentrations and incubation times that were experimentally optimized for each cell model for maximal uptake of NPs (see Text S1). After removing unbound NPs, the accumulation of gold NPs in individual cells was imaged and measured through gold NP-specific optical scattering (Figure 3a). Similar to previous experiments, we measured cell-averaged levels of scattering image amplitudes in target and non-target cells (Figure 4 row a). In all six cases we observed a higher level of NP signals in target cells, but all non-target cells also showed a significant level of NP uptake and formation of NP clusters (Figure 3a, 4a) so that the ratio of the NP signal for target versus non-target cells was below 10. However, higher pixel image amplitudes in target cells indicated the formation of the largest NP clusters in target cells.

**Figure 3:** Images and signals of gold NPs and PNBs in co-culture of target (HN31, labeled with Green Fluorescent Protein for identification) and non-target (NOM9) cells identically treated with 60 nm gold NSP-C225 conjugates (specific to EGFR that is overexpressed in target cells). A: overlay of bright field, fluorescent and scattering images shows target cells (green) and gold NPs (red) that can be found in both types of cells (the arrows show NP clusters in non-target cells); B: time-resolved scattering image of the same field shows PNB images (bright white spots) only in target cells; C,D: optical scattering time-responses of individual target (C) and non-target (D) cells show the PNB-specific signal only for target cell and the definition of the PNB lifetime of PNBs; time is measured from the moment of the exposure to the excitation laser pulse.

**Figure 4:** Cell population-averaged levels of optical scattering signals obtained for individual target (solid bar) and non-target (hollow bar) cells in six cell models represented by target/non-target cells/molecular targets: Squamous cell carcinoma, HN31/NOM9/EGFR (treated with 50 nm NS-Panitumumab conjugates); Lung cancer, A549/Fibroblast/EGFR (treated with 60 nm NSP-C225 conjugates); Epithelial cancer, HES/HS5/MUC1 (treated with 60 nm NSP-214D4 conjugates); Prostate cancer, C2-4B/HS5/PSMA (treated with 60 nm NSP-anti-PSMA conjugates); Leukemia, J32/JRT3-T3.5/CD3 and human T-cells, T-cell/BM/CD3 (treated with 60 nm NSP-OKT3 conjugates) for: Row A (red): gold NP amplitude of scattering image of gold NPs (a metric for the uptake of NPs by cells; Row B (purple): time-resolved scattering image amplitudes of PNBs; Row C (blue): PNB lifetimes. The ratio of the signals for target/non-target cell is shown for each parameter and cell model and indicates the cellular specificity of NPs (row A) and PNBs (rows B,C).

Next, target and non-target cells were identically treated with single laser pulses within the range of pulse fluences for PNB generation around NP clusters. For each cell model we experimentally determined the level of excitation pulse fluence that provided the generation of PNBs mainly in target cells and did not induce PNBs in non-target cells (Figure 3 b,c,d). The optical scattering images and time responses of individual cells were processed to compare the corresponding metrics for NP accumulation (Figure 4, row a) and PNB generation (Figure 4, row b,c) in target and non-target cells. Compared to NP signals, the PNB signals showed a much higher discrimination between target and non-target cells in all six. Cellular specificity of NPs and PNB was quantitatively shown through the ratios of the target cell signals to the corresponding signals in non-target cells (shown as colored numbers in each frame of Figure 4). Compared to NPs, the PNBs improved cellular specificity in some models by more than one order of magnitude. While the non-target cells showed significant uptake of NPs and even their potential aggregation into small clusters, no PNBs, or very small ones, were observed in non-target cells under identical treatment conditions (Figures 3 and 4).

The difference in cellular specificity of NPs and PNBs can be clearly seen in experiments with a co-culture of target (labeled with green fluorescent protein for identification) and non-target cells (Figure 3). At a specific fluence of the excitation laser pulse (25 mJ/cm^2^ at 778 nm) only target cells yielded PNBs while even adjacent non-target cells with gold NPs did not. Such a difference between NP and PNB signals was observed for all six cell models: adherent (HN31, HES, A549) and suspension (C4-2B, T-cells, Jurkat) cells, and for all molecular targets: receptors (EGFR, CD3, PSMA) and glycoproteins (MUC1). These results indicate the universal nature of the high cellular specificity of PNBs compared to that of gold NPs. Therefore, PNB provided better discrimination between target and non-target cells even when such cells were heterogeneously mixed.

### 3. Effects of the NP targeting vectors on the PNBs

The results reported above were obtained by using one type of antibody that was specific for the target cell in each cell model. In order to determine the role of the targeting vector in cellular specificity of PNBs, we completed three additional experiments in which the cellular specificity of NPs and PNBs was obtained for target (HN31) and non-target (cells) as a function of the targeting vector.

The first experiment compared NP and PNB signals for identical NPs with and without target-specific antibody (active vs passive targeting). We incubated cells identically with bare gold 60 nm spheres and with the conjugates of the same spheres to Panitumumab antibody that is specific against EGFR. The conditions of NP treatment were identical to those in Figure 4 and the laser treatment (532 nm, single pulse, 60 mJ/cm^2^) was identical for all cells. We observed no PNBs at all in target and non-target cells treated with “bare” NPs (Figure 5a) despite using an optical fluence that was above the PNB generation threshold even for the smallest clusters, but was below the PNB threshold for single NPs (Figure 2a). NP scattering amplitudes of both types of cells were comparable to those of the background scattering of intact cells. At the same time the cells treated with NP-Panitumumab conjugates (Figure 5a) returned a result similar to that observed earlier (Figure 4). PNB lifetime demonstrated a much higher contrast between target and non-target cells compared to scattering amplitudes measured for NPs. This experiment demonstrated that the important contribution of the targeting vector to NP uptake. The use of bare, non-conjugated NPs under the same targeting conditions (NP concentration and incubation time) was insufficient for achieving detectable NP effects.

**Figure 5:** Influence of targeting vectors on NP scattering amplitude (red) and PNB lifetime (blue) in individual target (solid bars) and non-target (hollow bars) cells. A: Target (HN31) and non-target (NOM9) cells identically treated with bare 60 nm gold NSPs and NSP-Panitumumab conjugates (antibody specific to EGFR that is overexpressed in HN31 cells); B: Effects of EGFR-specific antibodies C225 and Panitumumab as targeting vectors in HN31 cell model show 5 different combinations of the two antibodies; C: Effects of single and dual targeting antibodies against PSMA and EGFR (C225) in C4-2B cell model applied in combination with dual simultaneous optical excitation (so called rainbow PNB method) show synergistic enhancement of PNB lifetime in the rainbow mode.

The second experiment analyzed the effect of two anti-EGFR antibodies on NP and PNB signals for the same cell model of target (HN31) cells (Figure 5b). We applied two different antibodies, C225 and Panitumumab, that were separately conjugated to identical NPs (60 nm gold spheres). NPs were targeted in the following combinations that used identical concentrations of NPs and incubation times (Figure 5b). These combinations were (1) NP-C225, (2) NP-Panitumumab, (3) sequential targeting with Panitumumab alone and then with NP-C225, (4) sequential targeting with C225 alone and then NP-Panitumumab conjugates and (5) joint targeting of NP-C225 and NP-Panitumumab conjugates. NPs in cells were measured with NP-specific optical scattering amplitudes and the PNBs were characterized in the same cells with their lifetime measured under identical laser exposure to a single pulse (532 nm, 60 mJ/cm^2^) (Figure 5b). As can be seen from the data in Figure 5b, the PNB response to the variation of targeting conditions is more sensitive than that of NPs, whose uptake did not vary significantly. In particular, NSP-Panitumumab conjugate alone provided maximal PNB generation efficacy compared to all other combinations. Pre-treatment of the cells with free antibodies reduced the efficacy of PNB generation (lower lifetime) to possible blocking of EGFR with the administered free antibody during pre-treatment and, as a result, reduced uptake of NPs. It is interesting to note that the joint targeting of both NP conjugates also reduced the efficacy of PNB generation compared to Panitumumab alone (Figure 5b). This experiment demonstrated the superior sensitivity of PNBs compared to NPs to the targeting vector.

Finally, we compared the PNBs and NPs under the simultaneous combinatorial action of the two antibodies, each conjugated to a different NP type. This experiment employed the “rainbow” method of PNB generation which we recently developed [63], [80]. The method involves two different types of NPs being mixed in one cluster and simultaneously excited with two different laser pulses. We used the cell model of C4-2B cells described above. Gold nanospheres (NSP) of 60 nm, PNB excitation peak at 532 nm, and silica-gold nanoshells (NS) of 110 nm, PNB excitation peak at 787 nm, were conjugated to target-specific antibodies against PSMA [81] and non-specific antibody against EGFR (C225) as NSP-PSMA (spheres) and NS-C225 (shells), respectively. The target cells were incubated in three different combinations using identical nanoparticle concentration and incubation time. These combinations were (1) NSP-PSMA, (2) NS-C225 and (3) simultaneously with both conjugates. The uptake of all NPs was measured in individual cells through optical scattering for the three cases and did not show a significant difference (Figure 5c). PNBs were generated with two different simultaneous laser pulses of the same fluence of 38 mJ/cm^2^, each pulse wavelength matching the peak wavelengths of NSP and NS, respectively. In case 1, a single pulse was applied at 532 nm, in case 2 a single pulse was applied at 787 nm and in case 3 the two pulses, 532 nm and 787 nm, were simultaneously applied (Figure 5c). The laser fluence levels were adjusted to detect small PNBs in any of the three cases. Under such settings we detected similar small PNBs for cases 1 and 2 that employed one type of NP and one wavelength for optical excitation. However, in case 3, the PNB generated with the rainbow method showed a significant (about 10-fold) increase in the PNB lifetime compared to cases 1 and 2, which was much higher than the corresponding difference in NP scattering. The latter did not differ much for all three cases (Figure 5c). The PNB signal in case 3 apparently showed a synergistic enhancement of the PNB compared to cases 1 and 2, and even compared to the results presented above (Figure 4). Compared to Figure 4 (C4-2B cell, PNB lifetime) we increased the PNB lifetime with the rainbow mechanism by almost one order of magnitude, while at the same time reducing the laser fluence from 60 mJ/cm^2^ (Figure 4 for PSMA target) to 38 mJ/cm^2^. This was achieved through the simultaneous excitation of the two different plasmon resonances in co-localized NPs of two different types, NSP and NS. These were mixed in one cluster and simultaneously received two laser excitation pulses in the rainbow mode of PNB generation (details of the rainbow PNB method can be found in [63], [80]).

The three experiments described above demonstrate the role of NP targeting vectors in PNB generation. Depending on the vector employed, the PNBs varied from zero (for non-specific uptake of bare NPs) to the synergistic enhancement of the PNB in the rainbow mode.

## Discussion

### 1. Mechanism of cellular specificity of PNBs

As can be seen from Figure 4, the PNB method can better discriminate between target and non-target cells compared to NPs. Cellular specificity of PNBs was more than one order of magnitude higher than that of NPs (this can be clearly seen by comparing the ratios of the corresponding signals for target and non-target cells). Such an effect was achieved through the cluster-threshold mechanism of PNBs that prevents the generation of PNBs around non-specifically targeted single NPs (and their small clusters). This is due to the dependence of the PNB threshold upon cluster size and the low optical fluence applied. Since a similar effect of PNB specificity was observed in the 6 different cell models and for the different molecular targets we conclude that the mechanism of such high specificity should be universal and can be applied to many other cell targets that express specific molecules. The universal nature of PNB specificity can be explained by (1) the threshold mechanism of PNB generation, (2) the dependence of the PNB generation threshold fluence upon the size of the NP cluster (Figure 2) and (3) the universal mechanism of NP clustering through receptor-mediated endocytosis [38], [39], [49]. The latter is responsible for the maximal size of the cluster that determines the minimal PNB threshold fluence (Figure 2a) and other parameters (Figure 2b) of a PNB generated in a cell targeted with NPs. Since NP clustering is a result of endocytotic internalization and concentrating of NPs into a cluster, this is a universal mechanism for any living cell. The size of NP cluster in a cell and its ability to generate the PNB depends upon several factors:

#### 1.1. Targeting activity of NPs

Comparing NP and PNB signals in target (HN31) and non-target (NOM9) cells after active targeting with NP-Panitumumab conjugates (Figure 4) and passive targeting with “bare” identical NPs (Figure 5a) obtained under identical NP concentrations, incubation time and laser parameters, we concluded that the interaction of the targeting vector with specific cellular receptor is very important. The fact that passive targeting of both target and non-target cells returned no PNBs and the level of NP scattering was close to that of background means that the accumulation of bare non-conjugated NPs was very low and even endocytosis could not form a significant cluster due to the presumably low number of NPs accumulated at the cellular membrane. This assumption is fully in line with our previous data [39], [49] where we studied in detail the difference in cellular uptake of conjugated and bare gold NPs. These previous studies were performed only for one type of cell (only target cells were incubated without the comparison with non-target cells) and they directly showed a 10–100 fold reduction in the uptake of bare NPs [64] and a 20–80 fold increase in PNB generation threshold fluence compared to the same cells treated with conjugated NPs [38], [39]. Therefore, the combination of a sufficient number of specific receptors (typical for target cells) with NP vectors (active targeting) provides a maximal initial level of gold NPs accumulated at the cellular membrane.

#### 1.2. Activity of endocytosis

Endocytosis works as a universal process that takes NPs from the cellular membrane and concentrates them into clusters in the endo-lysosomal system. Due to the well-known safety of the formation of clusters of gold NPs, this is a relatively safe process providing that such NPs do not carry any toxic molecules [12], [38]–[46]. Our previous studies showed a significant reduction in NP cluster size and a decrease in PNB signals in target cells in response to the suppression of endocytosis in cells that accumulated a sufficient amount of gold NPs at their membranes [49].

Therefore, the size of the NP cluster built by a cell depends upon the activity of the clustering process (endocytosis) and the amount of NPs available at the cellular membrane. This mechanism does not prevent the formation of NP clusters in non-target cells, as we observed in our experiments (Figure 4, row a), and we found that this is a general rule. However, we also observed that non-target cells could not build as large NP clusters as target cells (Figure 4, row a) and, therefore, the mechanism of formation of the largest NP clusters (as PNB sources) is target cell-specific. By adjusting the laser fluence to the level matching the largest NP clusters (as demonstrated in Figure 2a and b) we provided the generation of PNBs only around the largest NP clusters associated with target cells. At the same time this fluence was not sufficient to generate PNB in non-target cells regardless the formation of small NP clusters. This principle is directly demonstrated by Figure 2b and it explains the much higher cellular specificity of PNB compared to the receptor-mediated active targeting of NPs. In many cases we observed only one PNB per target cell. This assumes the formation of at least one large NP cluster that was earlier found to be sufficient to support diagnostic and therapeutic functions of PNB (see the next section).

Based upon our previous findings we may estimate the size of NP clusters in the range of 5–100 NPs or 100–600 nm (for NPs with the diameter 50–60 nm) [39], [64]. Therefore, we conclude that the PNB is a universal mechanism for discriminating between target and non-target cells that demonstrates much higher specificity compared to that of NP targeting and can be considered as a universal solution for overcoming unwanted effects of non-specific cellular uptake of NPs.

### 2. Feasibility of PNBs for medicine

The high cellular specificity of any nano-agent makes sense only providing that such an agent can support the required biomedical functions. While the study of the biomedical effects of PNBs is outside the scope of this work, we may point out several cell-level effects observed earlier. We recently demonstrated *in vitro* and *in vivo* how optical, acoustical and mechanical localized tunable impacts of PNBs support five biomedical functions that are determined by the maximal size of the PNB which, in turn, is precisely controlled through the fluence of the laser pulse. These functions are diagnostics [40], [56], [57], [82], delivery of intracellular and extracellular molecular cargo [59]–[62], mechanical destruction of target cells [38], [40], [49], [57], [61], [63], [64], microsurgery [64], [65] and theranostics (the method that unites diagnosis, treatment and guidance of the treatment in one connected procedure) [40], [57], [63], [80]. All these functions were activated on demand and realized with cell selectivity with a single laser pulse of specific fluence, wavelength and duration. Such a short activation mechanism allows the reduction of the duration of the biomedical procedures to nano- and micro-seconds. In addition, we observed that the generation of even a single PNB in the target cell was sufficient to achieve the desired biomedical effect. This required a single NP cluster with a maximum of 100 particles. Therefore, the PNB mechanism provides a significant reduction of the NP load by several orders of magnitude, compared to other diagnostic and therapeutic methods based on gold NPs [1]–[7], [11], [20]–[29], [83]–[90]. The clustering mechanism of NPs considered above is not limited to endocytosis and may also employ the capability of NPs to self-assemble in various structures under specific conditions including NP clustering at the cellular membrane due to the co-localization of the receptors, fusion of endosomes and other chemical and biological mechanisms [91]. The combinatorial use of NP targeting vectors (defined in many labs) with the rainbow mechanism of PNBs [63], [80] provides the potential for a further improvement in specificity of the PNB effect in the complex biological environment of the human body. In addition, the PNB mechanism can be generalized to other types of non-gold NPs by co-localizing gold NPs (as PNB sources) with other NPs (such as drug carriers, for example). Recently we demonstrated how the intracellular delivery of the commercially available anti-cancer drug, doxorubicin liposomes (Doxil), can be improved through the mixed administration and clustering of gold NPs with Doxil and the intracellular release of the drug with co-localized PNBs [62].

In summary, we demonstrated that the specificity of the optical activation of nanoparticles in target cells can be improved by more than one order of magnitude through the threshold mechanism of plasmonic nanobubbles (PNBs). Due to its threshold nature the PNB method effectively discriminates between target and non-target cells under the identical treatment of both with nanoparticles and optical radiation. By combining the threshold nature of PNBs and the enhanced accumulation and clustering of nanoparticles in target cells, we showed that PNBs, unlike nanoparticles, can be minimized or totally avoided in non-target cells despite the uncontrollable non-specific uptake of nanoparticles by such cells. The PNB method will be compatible with many existing nanomedicine technologies in development, and will significantly improve their precision and selectivity.

## Supporting Information

Text S1 The detailed descriptions of cell models and the methods of plasmonic nanobubbles generation and detection.
(DOCX)

Figure S1 The expression level of EGFR in HN31 (cancer) and NOM9 (normal) cells as measured with Western blot method.
(TIF)

Figure S2 The expression level of CD3 receptor in human T-cells in the two cell samples of the peripheral blood mononuclear cells, target (CD3+) and non-target (CD3−) cells (the samples were stained with CD3-PE and analyzed on a Gallios Flow Cytometer from Beckman Coulter, Brea, CA).
(TIF)

Figure S3 Experimental scheme for plasmonic nanobubble (PNB) generation and detection: single gold NP clusters or individual cells in the sample chamber were mounted on the stage of inverted optical microscope; PNB generation was provided by the pulsed pump laser; a pulsed probe laser provided time-resolved optical scattering imaging of PNBs and a continuous probe laser provided the monitoring of the PNB size through its time-response.
(TIF)
